The article "In Vitro Activity of Various Sulbactam Compounds and Piperacillin/Tazobactam against Clinical Isolates of Different Gram-Negative Bacteria" was retracted in 2023. Reasons: signs of a paper mill; suspected computer-generated content; unreliable results or conclusions; concerns about the data.

# *In Vitro* Activity of Various Sulbactam Compounds and Piperacillin/Tazobactam against Clinical Isolates of Different Gram-Negative Bacteria

**DOI:** 10.1155/2021/1175379

**Published:** 2021-11-25

**Authors:** Shunian Xiao, Chuyue Zhuo, Chao Zhuo

**Affiliations:** State Key Laboratory of Respiratory Disease, The First Affiliated Hospital of Guangzhou Medical University, Guangzhou 510000, China

## Abstract

To provide direction for clinical application and pharmaceutical exploitation, the *in vitro* activity of sulbactam compounds and PIP/TAZ 8 : 1 against clinical isolates of Gram-negative bacteria (GNB, *n* = 976) was evaluated according to Clinical and Laboratory Standards Institute (CLSI) 2019. By minimal inhibitory concentrations (MICs), the resistance rate of all GNB to AMP/SBT 2 : 1 (56.9-100%) was significantly higher than other drugs, except the resistance rate of *Acinetobacter baumannii* (*Aba*, *n* = 204) to piperacillin/tazobactam (PIP/TAZ 8 : 1, 78.4%) which was close to it (76.5%). Additionally, the resistance rate of *Aba* to other compounds except AMP/SBT 2 : 1 differed greatly, but that of *Klebsiella pneumonia* (*Kpn*, *n* = 205) varied rarely. In addition, *Escherichia coli* (*Eco*, *n* = 204) and *Kpn* demonstrated low and high resistance rates, respectively. Compared with cefoperazone/sulbactam (CPZ/SBT 2 : 1), PIP/TAZ 8 : 1 had advantage in anti-*Eco* (RR = 0.5and OR = 2.17) and anti-*Kpn* activity (RR = 0.88and OR = 1.27), while its activity against *Pseudomonas aeruginosa* (*Pae*: *n* = 194, RR = 0.91, and OR = 1.12), *Aba* (RR = 1.31 and OR = 0.41), and other Enterobacteriaceae (other *Ebc*: *n* = 169, RR = 1.40, and OR = 0.62) was not better than CPZ/SBT 2 : 1. Although it had advantage against *Eco* (RR = 0.60 and OR = 1.78), *Pae* (RR = 0.67 and OR = 1.63), and *Aba* (RR = 0.70 and OR = 2.05), the inhibition effect of piperacillin/sulbactam (PIP/SBT 2 : 1) against *Kpn* (RR = 0.94 and OR = 1.12) and other *Ebc* was just similar with CPZ/SBT 2 : 1 (RR = 0.93 and OR = 1.10). Furthermore, the anti-*Eco* (RR = 0.70 and OR = 1.50), anti-*Kpn* (RR = 0.89 and OR = 1.24), and anti-*Pae* (RR = 0.74 and OR = 1.46) activities of ceftazidime/sulbactam (CAZ/SBT 1 : 1) had a weak advantage, while its activity against *Aba* (RR = 0.94 and OR = 1.15) and other *Ebc* (RR = 0.79 and OR = 1.36) was just close to CPZ/SBT 2 : 1. Moreover, the inhibitory effect of PIP/SBT 1 : 1 against all tested clinical species was more active than CPZ/SBT 2 : 1, while that of CAZ/SBT 2 : 1 against all species of bacteria analyzed was weaker than the controls.

## 1. Introduction

The emergence of clinically resistant bacteria increases the difficulty of curing infectious diseases [1–3]. Data from the China Antimicrobial Resistance Surveillance System (CARSS) from October 2017 to September 2018 showed that the total number of bacteria that could be included in the analysis of bacterial resistance reached 3,234,372 after removing duplicate strains based on the principle of retaining the first strain of the same bacteria in the same patient, of which Gram-negative bacteria (GNB) accounted for the majority (70.6%) (NHC, 2019). Gram-negative bacteria (GNB) are one of the most important public health problems in the world due to the high resistance to antibiotics. These microorganisms have important clinical significance in hospitals because since patients in the intensive care unit (ICU) are at high risk and GNB cause high morbidity and mortality [4–6]. The *Escherichia coli* (*Eco*), *Klebsiella pneumonia* (*Kpn*), *Acinetobacter baumannii* (*Aba*), *Pseudomonas aeruginosa* (*Pae*), and other Enterobacteriaceae (*Ebc*) are prominent clinical isolates of GNB which are resistant to the extended-spectrum *β*-lactamase (ESBL) ([7–9].

The article "In Vitro Activity of Various Sulbactam Compounds and Piperacillin/Tazobactam against Clinical Isolates of Different Gram-Negative Bacteria" was retracted in 2023. Reasons: signs of a paper mill; suspected computer-generated content; unreliable results or conclusions; concerns about the data.

To overcome the resistance of *β*-lactamase, medical institutions gradually advocate combining the *β*-lactam antibiotics and *β*-lactamase inhibitors to improve their antimicrobial activity. From the Status Report on Antimicrobial Administration and Antimicrobial Resistance in China [8], the proportion of cephalosporins/enzyme inhibitors, penicillin/enzyme inhibitors, and other *β*-lactams in the main antimicrobial applications of general hospitals was not low in 2018 (12%, 8%, and 6%, respectively).

Due to their low toxicity, strong inhibitory activity, and high stability, tazobactam (TAZ) and sulbactam (SBT) are widely applied as *β*-lactamase inhibitors for the treatment of resistant microbial infections. The tazobactam/piperacillin (TAZ/PIP 8 : 1), one of the most widely used antibiotic compounds in clinical practice, had been on the market in many countries in the 1990s [10]. Besides, ampicillin/sulbactam (AMP/SBT 2 : 1) was the earliest marketed variety of compound antibiotics containing sulbactam [11]. At present, the usage of cefoperazone/sulbactam is the largest among all enzyme inhibitor compounds used clinically in China [8]. Although the period of piperacillin/sulbactam (PIP/SBT 2 : 1) applied as an antibacterial medicine is not long, its clinical application has gradually become prevalent [12]. Furthermore, ceftriaxone/sulbactam, cefotaxime/sulbactam, mezlocillin/sulbactam, amoxicillin/sulbactam, and other sulbactam compounds currently are universal commercial medicines in China. Meanwhile, cefuroxime sodium/sulbactam, ceftazidime/sulbactam, and other compound drugs are also under development.

The article "In Vitro Activity of Various Sulbactam Compounds and Piperacillin/Tazobactam against Clinical Isolates of Different Gram-Negative Bacteria" was retracted in 2023. Reasons: signs of a paper mill; suspected computer-generated content; unreliable results or conclusions; concerns about the data.

To provide direction for the clinical application and pharmaceutical exploitation of antibiotics, ampicillin/sulbactam (AMP/SBT 2 : 1), cefoperazone/sulbactam (CPZ/SBT 2 : 1), ceftazidime/sulbactam (CAZ/SBT 1 : 1 and 2 : 1), piperacillin/sulbactam (PIP/SBT 1 : 1 and 2 : 1), and piperacillin/tazobactam (PIP/TAZ 8 : 1) against clinical isolates were assessed in this research. Particularly, the relative intensity of their antibacterial activities was compared with each other, taking the resistance rate of CPZ/SBT 2 : 1 as the controls.

## 2. Materials and Methods

### 2.1. Bacterial Isolates

From January 2017 to June 2019, a total of 976 nonduplicate GBA isolates were collected from six tertiary hospitals which were included in CARSS. All clinical isolates were sent to the Guangzhou Institute of Respiratory Health (Guangdong, China) and Peking Union Medical College Hospital of the Chinese Academy of Medical Sciences (Beijing, China) to test their minimal inhibitory concentrations (MICs). Also, all strains were reidentified by VITEK automatic microbial analyzer (bioMerieux, Republic of France). American Tissue Culture Collection (ATCC) 27853 and ATCC 25922 were used as the quality controls.

### 2.2. Experimental Medicines

The AMP/SBT (2 : 1), CPZ/SBT (2 : 1), PIP/SBT (1 : 1 and 2 : 1), CAZ/SBT (1 : 1 and 2 : 1), PIP/TAZ (8 : 1), SBT, and TAZ were supplied by Xiangbei Wellman Pharmaceutical Co., Ltd. (Hunan, China).

### 2.3. Minimal Inhibitory Concentrations (MICs)

The MICs of clinical isolates were determined by micro broth dilution method which was advocated by the Clinical Laboratory Standards Institute (CLSI) in M07Ed11E [11]. During the test, the concentration of tazobactam was fixedly configured to 4 *μ*g/mL and sulbactam solution was obtained according to the specific ratio of its compounds. Also, the antibiotics were configured into twelve concentrations by the double dilution method (0.063~128 *μ*g/mL). Meanwhile, several colonies cultured fresh overnight were picked and their turbidity was adjusted to 0.5 MCF in Mueller-Hinton Broth (MHB) (BD Difco, China) with a turbidity meter. Then, the colonies were cultured at 35°C for 20 h and their MICs were recorded. The corresponding standard strains were used as quality controls for each test. All tests were performed twice and in triplicate.

### 2.4. Evaluation of Antimicrobial Activity

#### 2.4.1. Susceptibility Testing

According to CLSI criteria in M100Ed30E [13], the MICs were converted into three levels: susceptible (S), intermediate (I), and resistant (R) in a standard dosing regimen. The breakpoint of susceptibility for the main ingredient of the medicine was used when the compounds did not have a breakpoint. Besides, if some special strains also lacked breakpoints of the main ingredient in standard dosing regimen in a single medicine, their breakpoints of Enterobacteriaceae to this medicine would be adopted.

The article "In Vitro Activity of Various Sulbactam Compounds and Piperacillin/Tazobactam against Clinical Isolates of Different Gram-Negative Bacteria" was retracted in 2023. Reasons: signs of a paper mill; suspected computer-generated content; unreliable results or conclusions; concerns about the data.

#### 2.4.2. Evaluation of Cross-Resistance

The AMP/SBT 2 : 1 was not analyzed when cross-resistance was assessed. The common sensitive rate and complete cross-resistant rate were, respectively, defined as the percentages of strains that were susceptible and resistant to the tested compounds, while the partial cross-resistant rate referred to the percentage of strains that were resistant to more than one medicine and were susceptible to one of them.

#### 2.4.3. Comparison of Antimicrobial Activity among Different Compounds

The resistance rate of clinical isolates to CPZ/SBT 2 : 1 was taken as the control. The susceptibility levels (S, I, or R) of different strains to various compounds were counted and converted into bidirectional ordinal R×C data with the same attributes. Subsequently, the consistency of the susceptibility between two compounds was analyzed by Kappa coefficient and their difference was assessed by McNemar's *x*^2^ test. When the susceptibility of the two compounds was significantly different (*p* < 0.05), the following items were evaluated to analyze their relative antimicrobial activity. The consistency of susceptibility was graded where their Kappa coefficients were in the ranges of 0.0-0.20, 0.21-0.40, 0.41-0.60, 0.61-0.80, and 0.81-1 which indicated that the consistency between the two compounds was extremely low, general, medium, highly similar, and almost identical, respectively. The ratio of resistance rate between the tested compounds and the controls was defined as the rate ratio (RR). 0.9-1.0, 0.7-0.8, 0.4-0.6, 0.1-0.3, and less than 0.1 represented that their advantage on RR was none, weak, medium, obvious, and extremely significant, respectively. Odds ratio (OR) = (number of resistant strains to the tested compounds × number of strains without resistance to the controls)/(number of strains without resistance to the tested compounds × number of resistant strains to the controls). 1.0-1.1, 1.2-1.4, 1.5-2.9, 3.0-9.0, and greater than 10 showed that their advantages on OR were none, weak, medium, obvious, and extremely significant, respectively. The difference in the resistance rate between the controls and the tested compounds was expressed as the attribution risk (AR). Attributable risk percent (ARP, %) = (AR/resistant rate of the controls) × 100% [14, 15].

## 3. Results

### 3.1. Distribution of Clinical Isolates

A total of 976 clinical isolates were collected, and their distributions of gender, age, specimens, and hospital departments are shown in Table 1. Other Enterobacteriaceae included *Enterobacter cloacae*, *Enterobacter aerogenes*, *Morganella morganii*, *Stenotrophomonas maltophilia*, *Serratia marcescens*, *Salmonella*, and *Proteus mirabilis*. Other specimens were consisted of amniotic fluid, pus, drainage fluid, ascites, bile, puncture fluid, bronchoalveolar lavage fluid, etc. Internal medicine contained general internal medicine, comprehensive internal medicine, hematology, fever ward, emergency observation ward, cardiology, neurology, gastroenterology, cardiovascular medicine, rheumatology and immunology, medical genetics, endocrinology, nephrology, respiratory medicine, infection control, etc. Surgery was composed of general surgery, orthopedics, urology, anorectal surgery, biliopancreatic surgery, gastrointestinal surgery, acupuncture and moxibustion, oral and maxillofacial surgery, interventional oncology, interventional radiology, urology, vascular surgery, hepatology, gastroenterology, pediatric surgery, surgical clinic, organ transplantation, neurosurgery, etc. Comprehensive clinics encompassed emergency general wards, geriatrics, general wards, gynecology, obstetrics, oncology, rehabilitation, neonatology, pediatrics, etc.

The article "In Vitro Activity of Various Sulbactam Compounds and Piperacillin/Tazobactam against Clinical Isolates of Different Gram-Negative Bacteria" was retracted in 2023. Reasons: signs of a paper mill; suspected computer-generated content; unreliable results or conclusions; concerns about the data.

From Table 1, the proportions of strains collected from male and female patients were similar. Also, most of the strains were collected from adults (41.44-44.31%) and elders (51.27-55.98%), but less for children (<5%). Besides, *Eco* was mostly derived from blood specimens, followed by the urinary system, and most of them were clinically isolated from the comprehensive clinic. Meanwhile, majorities of *Kpn*, *Aba*, *Pae*, and other *Ebc* were derived from the respiratory. Additionally, the amount of these strains isolated from the intensive care unit (ICU) and the comprehensive clinic was more than that of the internal medicine and surgery.

### 3.2. Evaluation of Antimicrobial Activity

#### 3.2.1. Resistance Rate

The resistance rate of different clinical isolates to various compounds is displayed in Figure 1. From Figure 1(a), various species of bacteria showed a high prevalence of resistance to AMP/SBT 2 : 1 (56.9%-100%). Moreover, the resistance rate of *Eco*, *Kpn*, *Aba*, *Pae*, and other *Ebc* to AMP/SBT 2 : 1 (*Eco*: 56.9%, *Kpn*: 72.2%, *Aba*: 76.5%, *Pae*: 100.0%, and other *Ebc*: 93.5%) was higher than that of CPZ/SBT 2 : 1 (*Eco*: 14.7%, *Kpn*: 48.8%, *Aba*: 59.6%, *Pae*: 23.7%, and other *Ebc*: 25.4%). Besides, the resistance rates of all species of bacteria to the remaining sulbactam compounds were as follows: CAZ/SBT 2 : 1 > CAZ/SBT 1 : 1 > PIP/SBT 2 : 1 > PIP/SBT 1 : 1. Among them, *Aba* has high resistance rates (>70%) to PIP/TAZ 8 : 1, CAZ/SBT 2 : 1, and AMP/SBT 2 : 1. Additionally, the resistance rates of the same clinical species to different compounds varied greatly except for *Aba*. The *Kpn* presented the highest resistance rate, followed by other *Ebc* and *Pae*, and *Eco* had the lowest resistance rate to the same compound. Furthermore, the resistance rate of *Aba* was also higher than that of *Eco*, *Pae*, and other *Ebc*, but its resistance rate to PIP/SBT 2 : 1 (41.9%) and PIP/SBT 1 : 1 (29.9%) was lower than that of *Kpn* (PIP/SBT 2 : 1 = 45.9%, PIP/SBT 1 : 1 = 41.5%). What is more, the resistance rate of the other four species of clinical isolates except for *Aba* to CPZ/SBT was higher than that of CAZ/SBT and their resistance rate to CAZ/SBT was also higher than that of PIP/SBT. Moreover, the resistance rate of five species of clinical isolates to CAZ/SBT 2 : 1 was all higher than CAZ/SBT 1 : 1 and their resistance rate to PIP/SBT 2 : 1 was also higher than PIP/SBT 1 : 1.

The article "In Vitro Activity of Various Sulbactam Compounds and Piperacillin/Tazobactam against Clinical Isolates of Different Gram-Negative Bacteria" was retracted in 2023. Reasons: signs of a paper mill; suspected computer-generated content; unreliable results or conclusions; concerns about the data.

From Figure 1(b) basing on the Wilcoxon rank sum test, GNB displayed the highest frequency of resistance to AMP/SBT 2 : 1 (rank sum = 34.0), but the lowest frequency of resistance to PIP/SBT 1 : 1 (rank sum = 6.0). The resistance rates of five species of clinical GNB to CAZ/SBT 1 : 1 (rank sum = 15.0) and PIP/SBT 2 : 1 (rank sum = 15.5) were close. Also, the resistance rates of them to PIP/TAZ 8 : 1 (rank sum = 20.0) and CAZ/SBT 2 : 1 (rank sum = 23.0) were similar.

#### 3.2.2. Cross-Resistance

The cross-resistance of various species of clinical isolates to PIP/SBT 2 : 1, CAZ/SBT 2 : 1, CAZ/SBT 1 : 1, PIP/SBT 1 : 1, CPZ/SBT 2 : 1, and PIP/TAZ 8 : 1 is exhibited in Figure 2. Six compounds had a high common sensitivity rate (about 50%), low complete cross-resistance rate (3.4~10.7%), and low partial cross-resistance rate to *Eco*, *Pae*, and other *Ebc*, which indicated that the therapeutic effects of these six compounds on the infections of *Eco*, *Pae*, and other *Ebc* could be replaced by each other. Furthermore, the common susceptibility rate of *Aba* to the six compounds was as low as 16.2% and its partial cross-resistance rate was up to 55.9%, representing that the susceptibility of the six compounds was highly variable. In addition, the common sensitivity rate, partial cross-resistance rate, and complete cross-resistance rate of *Kpn* to the six compounds were close (30~40%), denoting that the consistency of its sensitivity to these six compounds was high.

#### 3.2.3. Comparison of Antimicrobial Activity among Different Compounds

The statistical consistency, difference, and relative intensity of the resistance of *Eco*, *Kpn*, *Pae*, *Aba*, and other *Ebc* to different compounds are shown in Table 2. The resistance of various species to CPZ/SBT 2 : 1 was used as the controls. The Kappa coefficient of *Eco* for all the compounds was less than 0.2, which means that the consistency of its sensitivity was extremely low. Except for CAZ/SBT 2 : 1, the susceptibility of *Eco* between other compounds and CPZ/SBT 2 : 1 was significantly different (*p* < 0.05), where PIP/SBT 2 : 1 (RR = 0.60, OR = 1.78, AR = 5.88%, and ARP = 40.00%), PIP/SBT 1 : 1 (RR = 0.53, OR = 2.03, AR = 6.86%, and ARP = 46.67%), and PIP/TAZ 8 : 1 (RR = 0.50, OR = 2.17, AR = 7.35%, and ARP = 50.00%) had a medium advantage. However, CAZ/SBT 1 : 1 (RR = 0.70, OR = 1.50, AR = 4.41%, and ARP = 30.00%) was at a weak advantage compared to CPZ/SBT 2 : 1. Besides, the difference of *Eco* between CAZ/SBT 2 : 1 and CPZ/SBT 2 : 1 was not apparent (*p* = 0.106), and the consistency was also very low (Kappa coefficient < 0.2), suggesting that the antibacterial activities of these two compounds were complementary.

The article "In Vitro Activity of Various Sulbactam Compounds and Piperacillin/Tazobactam against Clinical Isolates of Different Gram-Negative Bacteria" was retracted in 2023. Reasons: signs of a paper mill; suspected computer-generated content; unreliable results or conclusions; concerns about the data.

Additionally, the susceptibility of *Kpn* to PIP/SBT 2 : 1 was generally consistent (Kappa coefficient = 0.227) and the difference in sensitivity between PIP/SBT 2 : 1 and CPZ/SBT 2 : 1 was visible (*p* = 9.43 × 10^−5^), but PIP/SBT 2 : 1 did not show an advantage (RR = 0.94, OR = 1.12, AR = 2.93%, and ARP = 6.00%). Moreover, the consistency in susceptibility of *Kpn* to other compounds except PIP/SBT 2 : 1 was extremely low (Kappa coefficient < 0.2) and the difference of *Kpn* between them to CPZ/SBT 2 : 1 was notable (*p* < 0.05), of which CAZ/SBT 1 : 1 (RR = 0.89, OR = 1.24, AR = 5.37%, and ARP = 11.00%), PIP/SBT 1 : 1 (RR = 0.85, OR = 1.34, AR = 7.32%, and ARP = 15.00%), and PIP/TAZ 8: 1 (RR = 0.88, OR = 1.27, AR = 5.85%, and ARP = 12.00%) had a weak advantage, but CAZ/SBT 2 : 1 (RR = 0.94, OR = 1.12, AR = 2.93%, and ARP = 6.00%) was nondominant.

Furthermore, the susceptibility of *Pae* to all compounds was remarkably low (Kappa coefficient < 0.2) and the difference of other medicines except PIP/TAZ 8 : 1 was obvious (*p* < 0.05) compared to CPZ/SBT 2 : 1, where PIP/SBT 1 : 1 (RR = 0.43, OR = 2.70, AR = 13.40%, and ARP = 56.52%) and PIP/SBT 2 : 1 (RR = 0.67, OR = 1.63, AR = 7.73%, and ARP = 32.61%) showed a moderate activity against *Pae*. The *Pae* also had a weak advantage in susceptibility to CAZ/SBT 1 : 1 (RR = 0.74, OR = 1.46, AR = 6.19%, and ARP = 26.09%), but with disadvantages to CAZ/SBT 2 : 1 (RR = 0.93, OR = 1.09, AR = 1.55%, and ARP = 6.52%).

What is more, the susceptibility of *Aba* between PIP/TAZ 8 : 1 and CPZ/SBT 2 : 1 was generally consistent (Kappa coefficient = 0.266) and their difference was noticeable (*p* = 2.09 × 10^−7^), but PIP/TAZ 8 : 1 was inferior (RR = 1.31, OR = 0.41, AR = −18.63%, and ARP = −31.15%). Also, the susceptibility of *Aba* was extremely low (Kappa coefficient < 0.2) to CAZ/SBT (1 : 1 and 2 : 1) and PIP/SBT (2 : 1 and 1 : 1), of which CAZ/SBT 1 : 1 is without an obvious difference (*p* = 0.0582) and CAZ/SBT 2 : 1 and PIP/SBT (2 : 1 and 1 : 1) with an apparent difference (*p* < 0.05). Among them, PIP/SBT 2 : 1 showed a weak advantage (RR = 0.70, OR = 2.05, AR = 17.73%, and ARP = 29.75%) and PIP/SBT 1 : 1 displayed a moderate advantage (RR = 0.50, OR = 3.49, AR = 29.90%, and ARP = 50.00%), but CAZ/SBT 2 : 1 was disadvantage (RR = 1.20, OR = 0.58, AR = −12.25%, and ARP = −20.49%).

The article "In Vitro Activity of Various Sulbactam Compounds and Piperacillin/Tazobactam against Clinical Isolates of Different Gram-Negative Bacteria" was retracted in 2023. Reasons: signs of a paper mill; suspected computer-generated content; unreliable results or conclusions; concerns about the data.

Besides, other *Ebc* had exceedingly low consistency of susceptibility to all compounds (Kappa coefficient < 0.2), and the statistical difference of CAZ/SBT 1 : 1, CAZ/SBT 2 : 1, and PIP/SBT 2 : 1 was not significant (*p* > 0.05) taking the resistance of CPZ/SBT 2 : 1 as controls. Although other *Ebc* had visible differences in resistance (*p* = 0.00350) between PIP/TAZ 8 : 1 and CPZ/SBT 2 : 1, PIP/TAZ 8 : 1 was at a disadvantage (RR = 1.40, OR = 0.62, AR = −10.06%, and ARP = −39.53%). In addition, other *Ebc* had notable differences in susceptibility between PIP/SBT 1 : 1 and CPZ/SBT 2 : 1, and the activity of PIP/SBT 1 : 1 was slightly superior to CPZ/SBT 2 : 1 (RR = 0.74, OR = 1.46, AR = 6.51%, and ARP = 25.58%).

## 4. Discussion

In this study, 976 clinical isolates of GNB were collected from six tertiary hospitals. Most of them were isolated from adult and elder patients, and the sex ratio of patients was close. Besides, the specimens were mainly blood, respiratory and urinary from the departments of ICU, internal medicine, surgery, and comprehensive clinic. Therefore, this research could provide a direction for the clinical treatment of bacterial infections in adults and elders, but it might not be extended to the infections in children.

Many types and proportions of SBT compounds had been marketed in China [8]. However, their antimicrobial activity and clinical advantages were not comprehensive for some of them were still under development. In this work, the resistance of five GNB to six SBT compounds and PIP/TAZ 8 : 1 was evaluated to provide direction for the clinical application and pharmaceutical exploitation of antibiotics. The assessment showed that the resistance rate of *Aba* to PIP/TAZ 8 : 1 (78.4%) was close to that of AMP/SBT 2 : 1 (76.5%). In addition, the resistance rate of *Eco*, *Kpn*, *Pae*, *Aba*, and other *Ebc* to AMP/SBT 2 : 1 was high (56.9~100%) and it was significantly higher than that to other compounds, indicating that AMP/SBT 2 : 1 was not recommended for the treatment of GNB infections in clinical practice. In recent years, the sensitivity of *Eco* to AMP/SBT 2 : 1 had also been decreasing, which was reported by lots of monitoring data [16, 17]. Besides, *Eco* was one of the most common pathogens causing intra-abdominal infections (IAIs), and AMP/SBT 2 : 1 might not be a good choice for the treatment of IAIs in patients with its resistant strains [18].

The article "In Vitro Activity of Various Sulbactam Compounds and Piperacillin/Tazobactam against Clinical Isolates of Different Gram-Negative Bacteria" was retracted in 2023. Reasons: signs of a paper mill; suspected computer-generated content; unreliable results or conclusions; concerns about the data.

Except for AMP/SBT 2 : 1, the analysis of the resistance rate and cross-resistance of other compounds showed that their susceptibility against *Aba* was quite different, suggesting that clinical medication should be selected based on the susceptibility of each medicine. Meanwhile, the difference in susceptibility of various compounds to *Kpn* was small, indicating that clinical isolates were likely to show resistance to another compound when they were resistant to others. Particularly, the resistance rate of *Eco* to five SBT compounds and PIP/TAZ 8 : 1 was low, which denoted that the compound analyzed still had clinical practicality against *Eco*.

Currently, CPZ/SBT 2 : 1 and PIP/TAZ 8 : 1 were the most often used antimicrobials in clinical practice in China (NHC, 2019). In this research, the statistical analysis was used to quantitatively evaluate the relative strength of the antimicrobial activity of six compounds except AMP/SBT 2 : 1 taking CPZ/SBT 2 : 1 as the controls. The evaluation presented that the inhibitory effect of PIP/SBT 1 : 1 against five GNB was better than CPZ/SBT 2 : 1. Besides, PIP/SBT 2 : 1 had better anti-*Eco*, anti-*Aba*, and anti-*Pae* activities, while its inhibitory effect to *Kpn* and other *Ebc* was analogous to CPZ/SBT 2 : 1. The inhibitory effect of CAZ/SBT 1 : 1 on the other three GNB had an advantage, but its antibacterial activity against *Abc* and other *Ebc* was just close to CPZ/SBT 2 : 1. But the inhibitory effect of CAZ/SBT 2 : 1 to four GNB except *Aba* was similar with CPZ/SBT 2 : 1 and its activity against *Aba* even was lower. In addition to the moderate advantage in the inhibition of *Eco* and the weak advantage in the inhibition of *Kpn*, the activity of PIP/TAZ 8 : 1 against *Aba* and other *Ebc* was at disadvantage.

Additionally, some previous studies indicated that increased dosage and prolonged infusion strategies should increase the possibility of obtaining germicidal exposure against GNB [19, 20]. Furthermore, combination therapy might be necessary when choosing empirical treatment, especially in *Aba* and *Kpn* which had the highest resistance rate, for many GNB had high antibiotic MICs in this study.

## 5. Conclusion

The antimicrobial activity of sulbactam compounds and PIP/TAZ 8 : 1 against GNB clinical isolates mainly isolated from the infected specimens of adults and elders was evaluated. The susceptibility test denoted that the resistance rate of AMP/SBT 2 : 1 was the highest, which was significantly higher than other SBT compounds. Besides, the activity of PIP/SBT (1 : 1 and 2 : 1) against clinically isolated GNB was better than or close to CPZ/SBT 2 : 1. Also, the antimicrobial activity of CAZ/SBT 1 : 1 was not inferior to CPZ/SBT 2 : 1 and that of CAZ/SBT 2 : 1 was not better than CPZ/SBT 2 : 1. The antibacterial activity of PIP/TAZ 8 : 1 against *Eco* and *Kpn* was better than CPZ/SBT 2 : 1, but its activity against *Aba* and other *Ebc* was inferior to CPZ/SBT 2 : 1. Furthermore, combination therapy might be necessary when choosing empirical treatment, especially in *Aba* and *Kpn* which had the highest resistance rate, for many GNB had high antibiotic MICs in this work.

The article "In Vitro Activity of Various Sulbactam Compounds and Piperacillin/Tazobactam against Clinical Isolates of Different Gram-Negative Bacteria" was retracted in 2023. Reasons: signs of a paper mill; suspected computer-generated content; unreliable results or conclusions; concerns about the data.

## Figures and Tables

**Figure 1:** The resistance rate of different clinical isolates to various compounds. (a) Resistance rate. (b) Wilcoxon rank. AMP/SBT: ampicillin/sulbactam; CPZ/SBT: cefoperazone/sulbactam; CAZ/SBT: ceftazidime/sulbactam; PIP/SBT: piperacillin/sulbactam; PIP/TAZ: piperacillin/tazobactam; *Eco*: *Escherichia coli*; *Kpn*: *Klebsiella pneumonia*; *Aba*: *Acinetobacter baumannii*; *Pae*: *Pseudomonas aeruginosa*; *Ebc*: Enterobacteriaceae.

**Figure 2:** The cross-resistance of various species of clinical isolates to PIP/SBT 2 : 1, CAZ/SBT 2 : 1, CAZ/SBT 1 : 1, PIP/SBT 1 : 1, PIP/SBT 1 : 1, CPZ/SBT 2 : 1, and PIP/TAZ 8 : 1. *Eco*: *Escherichia coli*, *n* = 204; *Kpn*: *Klebsiella pneumonia*, *n* = 205; *Aba*: *Acinetobacter baumannii*, *n* = 204; *Pae*: *Pseudomonas aeruginosa*, *n* = 194; *Ebc*: Enterobacteriaceae, *n* = 169.

**Table 1:** The distribution of clinical isolates to gender, age, specimens, and hospital departments.

Strains		*Eco*	*Kpn*	*Pae*	*Aba*	Other *Ebc*

Amounts		204	205	194	204	169

Male (%)		49.02	52.20	47.24	52.57	51.87

Age (%)	Children	2.94	3.90	2.58	4.41	3.78
	Adults	44.12	42.44	41.44	44.31	41.95
	Elders	52.94	53.66	55.98	51.27	54.27

Specimens (%)	Blood	58.33	23.41	8.25	9.80	11.24
	Respiratory	6.86	39.51	56.19	58.82	49.11
	Urinary	22.25	11.22	7.73	7.84	19.93
	Others	12.55	25.85	27.84	23.53	19.71

Departments (%)	Internal medicine	27.49	19.56	18.92	19.73	15.88
	Surgery	26.47	24.39	14.86	15.20	18.34
	ICU	14.27	26.34	28.56	34.06	31.16
	Comprehensive clinic	31.76	29.71	37.67	31.02	34.62

*Eco*: *Escherichia coli*; *Kpn*: *Klebsiella pneumonia*; *Aba*: *Acinetobacter baumannii*; *Pae*: *Pseudomonas aeruginosa*; ICU: intensive care unit; *Ebc*: Enterobacteriaceae.

The article "In Vitro Activity of Various Sulbactam Compounds and Piperacillin/Tazobactam against Clinical Isolates of Different Gram-Negative Bacteria" was retracted in 2023. Reasons: signs of a paper mill; suspected computer-generated content; unreliable results or conclusions; concerns about the data.

**Table 2:** The statistical consistency, difference, and relative intensity of the resistance of *Eco*, *Kpn*, *Pae*, *Aba*, and other *Ebc* to different compounds on the CPZ/SBT 2 : 1 as the control.

Isolates	Compounds	Resistance rate (%)	Cross-resistance rate (%)	Kappa coefficient	*p* values	RR	OR	AR (%)	ARP (%)
*Eco*	CAZ/SBT 1 : 1	10.3	7.35	0.0909	8.50 × 10^−4^	0.70^∗^	1.50^∗∗^	4.41	30.00
	CAZ/SBT 2 : 1	14.7	7.35	0.125	0.106	1.00	1.00	0.00	0.00
	PIP/SBT 1 : 1	7.8	5.39	0.157	0.00243	0.53^∗∗^	2.03^∗∗^	6.86	46.67
	PIP/SBT 2 : 1	8.8	7.35	0.125	0.0211	0.60^∗∗^	1.78^∗∗^	5.88	40.00
	PIP/TAZ 8 : 1	7.4	3.92	0.0735	1.71 × 10^−5^	0.50^∗∗^	2.17^∗∗^	7.35	50.00
*Kpn*	CAZ/SBT 1 : 1	43.4	41.46	0.157	5.10 × 10^−5^	0.89^∗^	1.24^∗^	5.37	11.00
	CAZ/SBT 2 : 1	45.9	42.44	0.0909	7.50 × 10^−5^	0.94	1.12	2.93	6.00
	PIP/SBT 1 : 1	41.5	40.49	0.191	1.34 × 10^−7^	0.85^∗^	1.34^∗^	7.32	15.00
	PIP/SBT 2 : 1	45.9	43.90	0.227^×^	0.0110	0.94	1.12	2.93	6.00
	PIP/TAZ 8 : 1	42.9	40.49	0.1250	5.03 × 10^−6^	0.88^∗^	1.27^∗^	5.85	12.00
*Pae*	CAZ/SBT 1 : 1	17.5	15.98	0.125	0.000457	0.74^∗^	1.46^∗^	6.19	26.09
	CAZ/SBT 2 : 1	22.2	18.56	0.157	0.00249	0.93	1.09	1.55	6.52
	PIP/SBT 1 : 1	10.3	10.31	0.157	3.00 × 10^−7^	0.43^∗∗^	2.70^∗∗^	13.40	56.52
	PIP/SBT 2 : 1	16.0	15.98	0.191	9.43 × 10^−5^	0.67^∗∗^	1.63^∗∗^	7.73	32.61
	PIP/TAZ 8 : 1	21.6	19.59	0.125	0.104	0.91	1.12	2.06	8.70
*Aba*	CAZ/SBT 1 : 1	56.4	53.43	0.0588	0.0582	0.94	1.15	3.43	5.74
	CAZ/SBT 2 : 1	72.1	56.37	0.0909	5.52 × 10^−6^	1.20	0.58	-12.25	-20.49
	PIP/SBT 1 : 1	29.9	29.41	0.157	<2.20 × 10^−16^	0.50^∗∗^	3.49^∗∗∗^	29.90	50.00
	PIP/SBT 2 : 1	41.9	40.89	0.0500	2.60 × 10^−7^	0.70^∗^	2.05^∗∗^	17.73	29.75
	PIP/TAZ 8 : 1	78.4	57.84	0.266	2.09 × 10^−7^	1.31	0.41	-18.63	-31.15
Other *Ebc*	CAZ/SBT 1 : 1	20.1	15.98	0.157	0.211	0.79	1.36	5.33	20.93
	CAZ/SBT 2 : 1	21.3	16.57	0.125	0.368	0.84	1.26	4.14	16.28
	PIP/SBT 1 : 1	18.9	18.34	0.157	0.0219	0.74^∗^	1.46^∗^	6.51	25.58
	PIP/SBT 2 : 1	23.7	21.89	0.157	0.0576	0.93	1.10	1.78	6.98
	PIP/TAZ 8 : 1	35.5	23.67	0.157	0.00350	1.40	0.62	-10.06	-39.53

The susceptibility of clinical isolates to CPZ/SBT 2 : 1 was used as the controls. The cross-resistance rate in the table was to analyze the cross-resistance of different clinical isolates between a specific compound and CPZ/SBT 2 : 1. The resistance rate of *Eco*, *Kpn*, *Aba*, *Pae*, and other *Ebc* to CPZ/SBT 2 : 1 was 14.7%, 48.8%, 23.7%, 59.6%, and 25.4%, respectively. The *p* > 0.05, 0.01 < *p* < 0.05, and *p* < 0.01 indicate that the difference was not significant, significant, and extremely significant, respectively. × represents that the sensitivity between this compound and CPZ/SBT 2 : 1 is generally consistent. ∗, ∗∗, and ∗∗∗ mean weak, medium, and obvious advantage, respectively. CPZ: cefoperazone; SBT: sulbactam; PIP: piperacillin; CAZ: ceftazidime; TAZ: tazobactam; RR: rate ratio; *p* values: significant difference; OR: odds ratio; AR: attributable risk; ARP: attributable risk percent; *Eco*: *Escherichia coli*, *n* = 204; *Kpn*: *Klebsiella pneumonia*, *n* = 205; *Aba*: *Acinetobacter baumannii*, *n* = 204; *Pae*: *Pseudomonas aeruginosa*, *n* = 194; *Ebc*: Enterobacteriaceae, *n* = 169.

The article "In Vitro Activity of Various Sulbactam Compounds and Piperacillin/Tazobactam against Clinical Isolates of Different Gram-Negative Bacteria" was retracted in 2023. Reasons: signs of a paper mill; suspected computer-generated content; unreliable results or conclusions; concerns about the data.

## Data Availability

The data used to support the findings of this study are currently under embargo while the research findings are commercialized. Requests for data, 12 months after publication of this article, will be considered by the corresponding author.
